The article "Scientific Evidence of Xuebijing Injection in the Treatment of Sepsis" was published in 2021. Journal: Evid Based Complement Alternat Med.

# Scientific Evidence of Xuebijing Injection in the Treatment of Sepsis

**DOI:** 10.1155/2021/6879278

**Published:** 2021-10-25

**Authors:** Sa Tian, Defang Qin, Yixuan Ye, Huawei Yang, Shuguang Chen, Tao Liu, Luming Hu, Huiming Li, Qian Niu, Xingzhan Zhang

**Affiliations:** Department of Intensive Care Unit, Guangdong Provincial Hospital of Chinese Medicine, Zhuhai, China

## Abstract

**Objectives:**

To systematically collate, appraise, and synthesize the current evidence on the Xuebijing injection (XBJI) for sepsis.

**Methods:**

Eight databases were searched for systematic reviews (SRs) or meta-analyses (MAs) on XBJI for sepsis. Assessing the Methodological Quality of Systematic Reviews-2 (AMSTAR-2), Preferred Reporting Item for Systematic Reviews and Meta-Analyses (PRISMA), and Grading of Recommendations, Assessment, Development, and Evaluation (GRADE) methods were used to assess the methodological quality, reporting quality, and evidence quality of the enrolled studies, respectively.

**Results:**

Out of the 13 studies that were included, all studies were rated critically low quality based on AMSTAR-2 results. Based on the results obtained from PRISMA, all studies were reported to be over 80%, while the GRADE system yielded three outcome measures rated high-quality, 16 were of moderate quality, and the rest were of low or critically low quality.

**Conclusions:**

The combination of XBJI and Western medicine (WM) showed significant synergy for the treatment of sepsis compared to WM alone. However, this conclusion should be treated with caution since the quality of the SRs/MAs providing the evidence was relatively low.

## 1. Introduction

Sepsis is a severe complication resulting from severe infection, severe trauma, burns, surgery, and shock. This complication is quite perilous, leading to septic shock and multiple organ dysfunction syndromes [1]. Sepsis is a common cause of death in the intensive care unit [2], where it accounts for one-third to one-half of hospital deaths [3], as more than six million people die from this disease worldwide each year [4]. Despite the major advances in antibiotics and supportive therapies over the last few decades, mortality from sepsis still maintains an increasing trend [5]. At present, there is still no effective treatment for sepsis. Conventional anti-infection and supportive therapies have also shown no significant improvement in the survival rate of patients with sepsis [6, 7]. Under these circumstances, complementary and alternative therapies have drawn attention.

Xuebijing injection (XBJI), a Chinese patent medicine, was developed by Professor Jinda Wang [8]. Professor Wang's work was based on the Xuefu Zhuyu decoction by Wang Qingren, a famous physician in the Qing dynasty. XBJI consists of five Chinese herbs (Radix Salviae, Carthami Flos, Chuanxiong Rhizoma, Angelicae Sinensis Radix, and Paeoniae Radix Alba) that contain approximately 30 bioactive compounds, such as hydroxysafflor yellow A, danshenol, ferulic acid, paeoniflorin, senna lactone I, and more [9]. The benefits of this medicine include detoxification and toning, elimination of bacteria and viruses, supplementation of vital energy, and improved blood circulation [9, 10]. In addition, the medicine can also inhibit the action of most inflammatory mediators and endotoxin, allowing the restoration of the immune response [11]. It was reported that XBJI can block the progression of sepsis through different mechanisms, such as antibacterial, antioxidative, and antiendotoxin [8, 11]. Therefore, XBJI has been approved as a State Category II New Drug for the treatment of sepsis in China and has been used in clinical practice [10]. Previous studies have shown that integrated medicine can reduce mortality due to sepsis [8], but the efficacy of XBJI combined with Western medicine (WM) still lacks scientific evidence. This study aims to systematically collate, appraise, and synthesize scientific evidence through the presentation of an overview of these SRs/MAs.

## 2. Methods

This study was registered in the PROSPERO registry (CRD42021264569). The methods of the Cochrane handbook and some high-quality reviews were followed [12, 13].

### 2.1. Strategy for Search

A systematic search was conducted utilizing PubMed, Cochrane Library, Embase, Web of Science, China National Knowledge Infrastructure, Chongqing VIP, SinoMed, and Wanfang databases from inception to June 2021. The following medical subject headings, terms, and relevant keywords were used in this search: Xuebijing, sepsis, and systematic review. The search strategies can be found in additional file 1.

### 2.2. Criteria of Inclusion and Exclusion

The studies that met the following criteria would be included for further evaluation. (1) Study type: participants enrolled in randomized controlled trials. (2) Subjects: patients diagnosed with sepsis according to internationally recognized diagnostic criteria. (3) Interventions: the experimental intervention was a combination of XBJI plus WM and the control intervention was WM alone. (4) Outcomes: one or more of the index of outcomes was present, such as 28-day mortality, acute physiology and chronic health evaluation (APACHE) II score, white blood cell, and procalcitonin (PCT). A study was excluded if it had the following factors: (1) it was a duplicate publication, (2) it was an expert comment or a conference report, (3) it did not undergo peer review, (4) the control group included XBJI, and (5) the lack of further data.

### 2.3. Literature Selection and Data Extraction

Two independent authors strictly followed the inclusion and exclusion criteria to conduct the study selection. Titles and abstracts of the literature were screened first, followed by the full text of all the initial qualified literature. The following data were extracted from each study: general information (first authors, country, and publication year), characteristics of the study (sample size and interventions), and results (outcomes and relative effect). A third author resolved any discrepancies between the two authors.

### 2.4. Quality Assessment

For the eligible studies that were included, two independent authors assessed the methodological quality, reporting quality, and evidence quality using the appraisal tool for systematic reviews of randomized and observational studies, Assessing the Methodological Quality of Systematic Reviews-2 (AMSTAR-2) [14], Preferred Reporting Item for Systematic Reviews and Meta-Analyses (PRISMA) [15], and Grading of Recommendations, Assessment, Development, and Evaluation (GRADE) [16], respectively. A third author resolved any discrepancies between the two authors. The items obtained from AMSTAR-2 and the checklists of PRISMA can be found in the additional file 2 and additional file 3.

## 3. Results

### 3.1. Results of the Literature Search

From the databases utilized, 132 articles were identified from the initial search. After 63 duplicate articles were removed, 69 were eliminated based on the title and abstract following the criteria. Then, the eligibility of the remaining 22 articles was evaluated by scanning the full text of each article. Finally, examining full text resulted in the exclusion of eight studies (Appendix file 4), and the remaining 14 studies [17–30] met the inclusion criteria. Flow diagram of the literature selection process is shown in Figure 1.

### 3.2. Basic Characteristics

The studies included were published between 2010 and 2021. Five of these reviews were published in English, while the remaining were in Chinese. The number of trials of the included reviews ranged from 11 to 49 studies, and the total number of subjects ranged from 399 to 1970. As for the intervention, all reviews compared XBJI plus WM as a treatment intervention, while the control group only utilized WM. Six reviews out of 13 applied the Jadad scale for methodological quality assessment of included trials, while the remaining seven reviews used the Cochrane criteria tool. Further details of the assessment are given in Table 1.

### 3.3. Quality Assessment

#### 3.3.1. Methodological Appraisal

The methodological quality was evaluated through AMSTAR-2. Among these studies, items 2, 4, 7, 9, 11, 13, and 15 were identified as key items. The key factors affecting the methodological quality were item 2 (no review established protocol), item 4 (11 reviews did not provide the search strategy), item 7 (no review provided a list of excluded trials), item 10 (6 reviews did not report the sources of funding), and item 16 (5 reviews did not report any potential sources of conflict of interest). Further details of this assessment are given in Table 2.

#### 3.3.2. Quality of Reporting Appraisal

The quality of reporting was evaluated using the PRISMA guidelines, which included 7 sections and 27 items. The sections of the studies, including project title, abstract, introductions, and discussion, were comprehensively reported (100%). In the Methods section, the protocol and registration numbers were not reported in any of the reviews (0%), while the searches were completely reported in three reviews (21.4%), and the additional analyses conducted in the studies were reported in 10 reviews (78.6%). In the results section, the additional analyses were reported in 8 reviews (57.1%). Furthermore, funding was only reported in 8 reviews (57.1%). Further details are given in Table 3.

#### 3.3.3. GRADE Evidence Quality Classification

The 13 reviews included 43 outcome indicators that were related to the effectiveness of XBJI for sepsis. Three outcomes were identified as high quality, 16 were identified to be of moderate quality, 19 were identified to be of low quality, and the remaining 3 were identified to be with critically low quality. The risk of bias, inconsistency, imprecision, and publication bias were the main reasons for the decrease in quality. Further details are given in Table 4.

### 3.4. Description of Efficacy

#### 3.4.1. Effect of the Interventions

The effects of the outcome indicators related to the effectiveness of XBJI for sepsis are given in Table 4. Twelve reviews [17, 24, 26, 27, 29, 30] reported the meta-analysis results of the 28-day mortality. The results revealed that the 28-day mortality rate of the XBJI group was lower when compared to the control group. Night reviews [17, 21, 23, 25, 27, 30] reported the outcomes for the APACHE II score revealed that XBJI combined with WM was superior to a single WM in improving the APACHE II score. Three reviews [17, 19, 20] then reported the outcomes for the duration of mechanical ventilation. These results showed that the time of mechanical ventilation of XBJI combined with the WM group was shorter than the control group, while three reviews [17, 19, 20] reported that the outcomes for the length of ICU stay showed that the XBJI plus WM group had an advantage over the WM only group in reducing the length of ICU stay. Two reviews [18, 20] reported the outcomes for body temperature changes, where their results revealed that XBJI accompanied with WM could lower body temperature better than the treatment with WM alone. Five reviews [17, 19, 21, 22, 25] then reported the serum levels of PCT for XBJI in combination with WM and the control group. The results showed that the XBJI plus WM group had a lower PCT level than the control group. Furthermore, four reviews [18, 25, 27, 28, 30] reported that the white blood cell count of the XBJI plus WM group was lower than the control group.

#### 3.4.2. Safety of the Interventions

A total of five reviews [18, 19, 24, 25, 29] mentioned the adverse effects of XBJI for sepsis. Wherein, no adverse effects were reported in 3 reviews [18, 24, 25]. Two reviews [19, 29] identified the following side effects, including pruritus and mild diarrhea, but no significant difference was found compared with the control group.

## 4. Discussion

The treatment of sepsis remains unsatisfactory despite the use of combined antibiotics and therapy [18]. Therefore, it is essential to identify a more effective, innovative, and adjunctive medicine for clinical application [17]. XBJI has been widely used for sepsis in clinical practices in China, wherein pharmacological experiments have demonstrated that it may be a promising treatment for sepsis. As the number of SRs/MAs regarding XBJI for sepsis has increased, scientific evidence for evidence-based medicine is still weak. Hence, we conducted this study to collate, appraise, and synthesize the evidence on XBJI systematically.

This overview summarized the scientific evidence on the effectiveness and safety of XBJI for sepsis by evaluating the methodological quality, reporting quality, and evidence quality of SRs/MAs. The current evidence indicated that subjects treated using the combination of XBJI and WM showed a significant reduction in the 28-day mortality, APACHE II score, duration of mechanical ventilation, length of ICU stays, body temperature, serum levels of PCT, and white blood cell count as compared to those treated with WM alone. However, this conclusion must be considered with caution, given the limitations of the study. According to the results of AMSTAR-2, all reviews failed to meet the key item of I2 (established protocol) and I7 (provided the list of excluded trials), which may contribute to the possibility of risk of bias and undermine the reliability of the conclusions. Then, according to the results of PRISMA, I5 (protocol and registration protocol and registration), I8 (search), I16 (additional analyses), I23 (additional analyses), and I27 (funding) were not reported adequately. This reasoning may increase the risk of bias and affect the rigor of SRs/MAs. Based on the results of GRADE, only three outcome indicators provided high-quality evidence, 16 provided moderate-quality evidence, and the remaining 24 provided low or critical low-quality evidence. These results indicate that the conclusions of the reviews may differ from the true results and therefore cannot be used as an evidence-based basis. Furthermore, it is worth noting that almost all the included SRs/MAs indicated that XBJI plus WM seems to have significant clinical efficacy in the therapy of patients with sepsis. However, most authors did not wish to draw definitive conclusions due to low methodological quality or the small size of the enrolled studies.

The pathogenesis of sepsis includes inflammation, immune dysregulation, and coagulopathy, with uncontrolled inflammation being the most critical for patients [31]. According to traditional Chinese medicine, the basic pathogenesis of sepsis involves the accumulation of toxins in the interior and extremities, leading to siltation, stagnation, and weakened body resistance [10]. XBJI was then created according to this theory as a possible treatment for sepsis [32]. XBJI was composed of five herbs containing approximately 30 bioactive compounds, including hydroxysafflor yellow A, danshenol, ferulic acid, paeoniflorin, and senna lactone I, among others [17]. Therefore, XBJI has the effects of “multiingredient, multitarget, and multipathway,” including detoxifying and toning, elimination of bacteria and viruses, supplementing vital energy, and invigorating blood circulation [19]. Modern pharmacological studies have uncovered the potential therapeutic mechanisms of XBJI for sepsis. It was reported that XBJI could regulate the immune status of the body by inhibiting the release of inflammatory mediators, reducing the total accumulation of endotoxins, bacterial toxin detoxification, and reducing the total amount of oxygen free radicals in the circulatory system. These effects help regulate the overall microcirculatory status of the body, protect and restore vascular endothelial function, and increase the total blood perfusion of the organs [19]. Moreover, XBJI also reduces the release of mast cells, which reduces the synthetic activity of fibroblasts. These effects lead to the avoidance of inflammatory exudation and increase the permeability of blood vessels [11]. Furthermore, XBJI helps the body absorb necrotic material and hematoma, promoting rehabilitation [33]. Thus, the use of XBJI is considered a promising approach for the treatment of sepsis.

To our knowledge, this is the first study to systematically collate, appraise, and synthesize the scientific evidence on XBJI for sepsis. However, we found that most of the included reviews were of poor quality, which could result in these studies having low credibility. Furthermore, the AMSTAR-2 tool, PRISMA checklist, and the GRADE system are highly subjective as different reviewers have their independent judgment. The subjectivity of the authors may then lead to varying results as subjective factors or errors cannot be eliminated.

## 5. Conclusion

The combination of XBJI and WM showed significant synergy for the treatment of sepsis compared to the use of WM alone. It provided a new and prospective therapeutic method for sepsis. However, this conclusion should be treated with caution as the quality of SRs/MAs providing evidence was generally low.

## Figures and Tables

**Figure 1:** Flow diagram of the literature selection process.

**Table 1:** Basic characteristics description.

Author, year	Country	Sample size	Treatment intervention	Control intervention	Quality assessment tool	Conclusion summary
Chen et al. [17] 2018	China	17 (1247)	XBJI + WM	WM	Cochrane criteria	The XBJI and ulinastatin combination therapy appeared to be more effective for the treatment of sepsis when compared with the use of ulinastatin alone.
Li et al. [18] 2018	China	16 (1144)	XBJI + WM	WM	Cochrane criteria	This study suggested that supplementation with XBJI in addition to the conventional treatment appeared to be more effective for the treatment of sepsis as compared to the conventional treatment alone.
Xiao et al. [19] 2018	China	16 (1335)	XBJI + WM	WM	Cochrane criteria	The combination therapy appeared to be more effective for the treatment of sepsis compared to the conventional treatment alone. It was also observed that the risk of adverse events did not increase.
Zheng et al. [20] 2018	China	16 (1192)	XBJI + WM	WM	Cochrane criteria	Our results found that XBJI when combined with ulinastatin was superior to both routine therapies and the single administration of either ulinastatin or XBJI.
Xiao et al. [21] 2017	China	49 (1801)	XBJI + WM	WM	Jadad	The combination therapy appeared to be more effective for the treatment of sepsis when compared to conventional treatment alone.
Liu et al. [22] 2021	China	16 (1423)	XBJI + WM	WM	Jadad	This study suggested that supplementation with XBJI in addition to the conventional treatment appeared to be more effective for the treatment of sepsis as compared to conventional treatment alone.
Zhang et al. [23] 2021	China	15 (930)	XBJI + WM	WM	Cochrane criteria	The utilization of XBJI has a certain effect on the improvement of the inflammatory response and increased level of platelets.
Zhou et al. [24] 2016	China	8 (399)	XBJI + WM	WM	Jadad	The homogeneity of the reduced mortality rate and the available evidence was sufficient to support the use of XBJI as adjunctive therapy for sepsis.
Li et al. [25] 2016	China	11 (803)	XBJI + WM	WM	Cochrane criteria	Clinical evidence showed that the addition of XBJI to the conventional treatment could improve the clinical efficacy in the treatment of sepsis.
Xu et al. [26] 2014	China	18 (1172)	XBJI + WM	WM	Jadad	The combined use of XBJI based on conventional treatment could improve the survival rate of patients with sepsis.
Li et al. [27] 2013	China	13 (1280)	XBJI + WM	WM	Jadad	XBJI had a certain effect in improving the inflammatory response and coagulation function in patients with sepsis. These effects reduced mortality and improved the APACHE II scores.
Sun et al. [28] 2012	China	18 (1080)	XBJI + WM	WM	Jadad	The existing results showed that the application of XBJI in the treatment of sepsis could significantly reduce the white blood cell count in the plasma of patients.
Hu et al, [29] 2010	China	25 (1970)	XBJI + WM	WM	Cochrane criteria	The evidence available showed that XBJI might decrease mortality, ineffectiveness, incidence of complication, and average hospital stay. It could also reduce the APACHE II score in patients with sepsis.
Wu et al. [30] 2020	China	14 (938)	XBJI + WM	WM	Cochrane criteria	XBJI can improve the clinical symptoms, significantly reduce the mortality, and has a high clinical application value.

**Table 2:** Result of methodological quality.

Reviews	AMSTAR-2																Quality
	I1	I2	I3	I4	I5	I6	I7	I8	I9	I10	I11	I12	I13	I14	I15	I16	
Chen et al. [17] 2018	Y	PY	Y	Y	Y	Y	N	Y	Y	Y	Y	Y	Y	Y	Y	Y	CL
Li et al. [18] 2018	Y	PY	Y	Y	Y	Y	N	Y	Y	Y	Y	Y	Y	Y	Y	Y	CL
Xiao et al. [19] 2018	Y	PY	Y	Y	Y	Y	N	Y	Y	Y	Y	Y	Y	Y	Y	Y	CL
Zheng et al. [20] 2018	Y	PY	Y	PY	Y	Y	N	Y	Y	Y	Y	Y	Y	Y	Y	Y	CL
Xiao et al. [21] 2017	Y	PY	Y	PY	Y	Y	N	Y	Y	Y	Y	Y	Y	Y	Y	Y	CL
Liu et al. [22] 2021	Y	PY	Y	PY	Y	Y	N	Y	Y	Y	Y	Y	Y	Y	Y	Y	CL
Zhang et al. [23] 2021	Y	PY	Y	PY	Y	Y	N	Y	Y	Y	Y	Y	Y	Y	Y	Y	CL
Zhou et al. [24] 2016	Y	PY	Y	PY	Y	Y	N	Y	Y	Y	Y	Y	Y	Y	Y	Y	CL
Li et al. [25] 2016	Y	PY	Y	PY	Y	Y	N	Y	Y	N	Y	Y	Y	Y	Y	N	CL
Xu et al. [26] 2014	Y	PY	Y	PY	Y	Y	N	Y	Y	N	Y	Y	Y	Y	Y	N	CL
Li et al. [27] 2013	Y	PY	Y	PY	Y	Y	N	Y	Y	N	Y	Y	Y	Y	Y	N	CL
Sun et al. [28] 2012	Y	PY	Y	PY	Y	Y	N	Y	Y	N	Y	Y	Y	Y	Y	N	CL
Hu et al. [29] 2010	Y	PY	Y	PY	Y	Y	N	Y	Y	N	Y	Y	Y	Y	Y	N	CL
Wu et al. [30] 2020	Y	PY	Y	PY	Y	Y	N	Y	Y	N	Y	Y	Y	Y	Y	Y	CL

**Table 3:** Result of reporting quality.

Items	Chen, 2018	Li, 2018	Xiao, 2018	Zheng, 2018	Xiao, 2017	Liu, 2021	Zhang, 2021	Zhou, 2016	Li, 2016	Xu, 2014	Li, 2014	Sun, 2012	Hu, 2010	Wu, 2020	Compliance (%)
# 1	Y	Y	Y	Y	Y	Y	Y	Y	Y	Y	Y	Y	Y	Y	100
# 2	Y	Y	Y	Y	Y	Y	Y	Y	Y	Y	Y	Y	Y	Y	100
# 3	Y	Y	Y	Y	Y	Y	Y	Y	Y	Y	Y	Y	Y	Y	100
# 4	Y	Y	Y	Y	Y	Y	Y	Y	Y	Y	Y	Y	Y	Y	100
# 5	N	N	N	N	N	N	N	N	N	N	N	N	N	N	0
# 6	Y	Y	Y	Y	Y	Y	Y	Y	Y	Y	Y	Y	Y	Y	100
# 7	Y	Y	Y	Y	Y	Y	Y	Y	Y	Y	Y	Y	Y	Y	100
# 8	Y	Y	Y	PY	PY	PY	PY	PY	PY	PY	PY	PY	PY	PY	21.4
# 9	Y	Y	Y	Y	Y	Y	Y	Y	Y	Y	Y	Y	Y	Y	100
# 10	Y	Y	Y	Y	Y	Y	Y	Y	Y	Y	Y	Y	Y	Y	100
# 11	Y	Y	Y	Y	Y	Y	Y	Y	Y	Y	Y	Y	Y	Y	100
# 12	Y	Y	Y	Y	Y	Y	Y	Y	Y	Y	Y	Y	Y	Y	100
# 13	Y	Y	Y	Y	Y	Y	Y	Y	Y	Y	Y	Y	Y	Y	100
# 14	Y	Y	Y	Y	Y	Y	Y	Y	Y	Y	Y	Y	Y	Y	100
# 15	Y	Y	Y	Y	Y	Y	Y	Y	Y	Y	Y	Y	Y	Y	100
# 16	Y	Y	Y	Y	Y	N	Y	Y	N	Y	Y	N	Y	Y	78.6
# 17	Y	Y	Y	Y	Y	Y	Y	Y	Y	Y	Y	Y	Y	Y	100
# 18	Y	Y	Y	Y	Y	Y	Y	Y	Y	Y	Y	Y	Y	Y	100
# 19	Y	Y	Y	Y	Y	Y	Y	Y	Y	Y	Y	Y	Y	Y	100
# 20	Y	Y	Y	Y	Y	Y	Y	Y	Y	Y	Y	Y	Y	Y	100
# 21	Y	Y	Y	Y	Y	Y	Y	Y	Y	Y	Y	Y	Y	Y	100
# 22	Y	Y	Y	Y	Y	Y	Y	Y	Y	Y	Y	Y	Y	Y	100
# 23	Y	Y	Y	Y	Y	N	N	Y	N	Y	Y	N	N	N	57.1
# 24	Y	Y	Y	Y	Y	Y	Y	Y	Y	Y	Y	Y	Y	Y	100
# 25	Y	Y	Y	Y	Y	Y	Y	Y	Y	Y	Y	Y	Y	Y	100
# 26	Y	Y	Y	Y	Y	Y	Y	Y	Y	Y	Y	Y	Y	Y	100
# 27	Y	Y	Y	Y	Y	Y	Y	Y	N	N	N	N	N	N	57.1

**Table 4:** Results of evidence quality.

Review	Outcomes	Certainty assessment						Relative effect (95% CI)	Quality
		Design	Limitations	Inconsistency	Indirectness	Imprecision	Publication bias		
Chen et al. [17] 2018	28 days mortality	Rct	No	No	No	No	No	RR 0.54 (0.39, 0.73)	⊕⊕⊕⊕⊕ high
	Duration of mechanical ventilation	Rct	No	No	No	No	No	SMD −1.13 (−1.30, −0.95)	⊕⊕⊕⊕⊕ high
	Length of ICU stay	Rct	No	No	No	No	No	SMD −0.84 (−1.00, −0.67)	⊕⊕⊕⊕⊕ high
	APACHE II score	Rct	No	Serious	No	No	No	SMD −1.09 (−1.49, −0.69)	⊕⊕⊕⊕○ moderate
	Serum levels of PCT	Rct	Serious	Serious	No	No	No	SMD −1.61 (−2.23, −0.98)	⊕⊕⊕○○ low

Li et al. [18] 2018	28 days mortality	Rct	Serious	No	No	No	No	RR 0.62 (0.51, 0.76)	⊕⊕⊕⊕○ moderate
	APACHE II score	Rct	Serious	Serious	No	No	No	MD = −3.51 (−4.49, −2.54)	⊕⊕⊕○○ low
	White blood count	Rct	Serious	Serious	No	Serious	Serious	MD = −8.00 (−10.18, −5.82)	⊕○○○○ very low
	Body temperature changes	Rct	Serious	No	No	No	No	MD = −0.43 (−0.55, −0.31)	⊕⊕⊕⊕○ moderate

Xiao et al. [19] 2018	Duration of mechanical ventilation	Rct	Serious	No	No	No	No	SMD −0.90 (−1.07, −0.72)	⊕⊕⊕⊕○ moderate
	Length of ICU stay	Rct	Serious	No	No	No	No	SMD −0.89 (−1.04, −0.73)	⊕⊕⊕⊕○ moderate
	28 days survival rate	Rct	Serious	No	No	No	No	RR 1.20 (1.08, 1.34)	⊕⊕⊕⊕○ moderate
	Serum levels of PCT	Rct	Serious	Serious	No	No	No	SMD −0.57 (−0.77, −0.38)	⊕⊕⊕○○ low
	APACHE II score	Rct	Serious	Serious	No	No	No	SMD −1.16 (−1.57, −0.75)	⊕⊕⊕○○ low

Zheng et al. [20] 2018	28 days mortality	Rct	Serious	No	No	No	No	RR 0.64 (0.43, 0.96)	⊕⊕⊕⊕○ moderate
	APACHE II score	Rct	Serious	Serious	No	No	No	SMD −1.21 (−1.62, −0.80)	⊕⊕⊕○○ low
	Duration of mechanical ventilation	Rct	Serious	Serious	No	No	No	SMD −1.04 (−1.40, −0.67)	⊕⊕⊕○○ low
	Length of ICU stay	Rct	Serious	No	No	No	No	SMD −0.83 (−1.03, −0.64)	⊕⊕⊕⊕○ moderate

Xiao et al. [21] 2017	28 days mortality	Rct	Serious	No	No	No	Serious	RR 0.51 (0.44, 0.59)	⊕⊕⊕○○ low
	APACHE II score	Rct	Serious	Serious	No	No	No	WMD −3.70 (−4.31, −3.09)	⊕⊕⊕○○ low
	Serum levels of PCT	Rct	Serious	Serious	No	No	No	WMD −1.26 (−1.63, −0.88)	⊕⊕⊕○○ low
	White blood count	Rct	Serious	Serious	No	No	No	WMD −1.48 (−2.03, −0.94)	⊕⊕⊕○○ low
	Body temperature changes	Rct	Serious	Serious	No	No	No	WMD −0.50 (−0.92, −0.07)	⊕⊕⊕○○ low

Liu et al. [22] 2021	28 days mortality	Rct	Serious	No	No	No	No	RR 1.20 (1.15, 1.25)	⊕⊕⊕⊕○ moderate
	White blood count	Rct	Serious	Serious	No	No	No	MD −1.95 (−3.62, −0.28)	⊕⊕⊕○○ low
	Serum levels of PCT	Rct	Serious	Serious	No	No	No	MD −1.29 (−1.97, −0.62)	⊕⊕⊕○○ low

Zhang et al. [23] 2021	28 days mortality	Rct	Serious	No	No	No	No	OR 0.52 (0.38, 0.71)	⊕⊕⊕⊕○ moderate
	APACHE II score	Rct	Serious	No	No	No	No	WMD −2.65 (−3.23, −2.08)	⊕⊕⊕⊕○ moderate

Zhou et al. [24] 2016	28 days mortality	Rct	Serious	No	No	Serious	No	RR 0.61 (0.41, 0.90)	⊕⊕⊕○○ low

Li et al. [25] 2016	Effective rate	Rct	Serious	No	No	No	No	OR 2.90 (1.89, 4.47)	⊕⊕⊕⊕○ moderate
	APACHE II score	Rct	Serious	No	No	No	No	MD −4.01 (−4.88, −3.13)	⊕⊕⊕⊕○ moderate
	White blood count	Rct	Serious	No	No	Serious	Serious	MD −4.31 (−6.73, −1.89)	⊕○○○○ very low
	Serum levels of PCT	Rct	Serious	No	No	Serious	Serious	MD −1.42 (−1.90, −0.95)	⊕○○○○ very low

Xu et al. [26] 2014	28 days survival rate	Rct	Serious	No	No	No	No	RR 1.21 (1.12, 1.29)	⊕⊕⊕⊕○ moderate

Li et al. [27] 2014	28 days mortality	Rct	Serious	No	No	No	No	OR 0.39 (0.27, 0.58)	⊕⊕⊕⊕○ moderate
	APACHE II score	Rct	Serious	Serious	No	No	No	WMD −3.43 (−4.72, −2.15)	⊕⊕⊕○○ low
	White blood count	Rct	Serious	No	No	Serious	Serious	WMD −2.94 (−3.49, −2.38	⊕○○○○ very low

Sun et al. [28] 2012	White blood count	Rct	Serious	Serious	No	No	No	WMD −1.87 (−2.92, −0.81)	⊕⊕⊕○○ low

Hu et al. [29] 2010	28 days mortality	Rct	Serious	Serious	No	No	No	RR 0.65 (0.54, 0.79)	⊕⊕⊕○○ low

Wu et al. [30] 2020	28 days mortality	Rct	Serious	No	No	No	No	RR 0.52 (0.40, 0.67)	⊕⊕⊕⊕○ moderate
	APACHE II score	Rct	Serious	Serious	No	No	No	MD −5.48 (−7.52, −3.43)	⊕⊕⊕○○ low
	White blood count	Rct	Serious	Serious	No	No	No	MD −2.26 (−3.35, −1.17)	⊕⊕⊕○○ low
	C-reactive protein	Rct	Serious	Serious	No	No	No	MD −37.43 (−56.70, −18.16)	⊕⊕⊕○○ low

ICU, intensive care unit; APACHE, acute physiology and chronic health evaluation; PCT, procalcitonin. RCT, randomized controlled trials; WMD, weighted mean difference; SMD, standard mean difference; MD, mean difference; OR, odds ratio; RR, relative risk.

## Data Availability

The data generated or analyzed during this study are included within this article.

## Abbreviations

XBJI: Xuebijing injection
WM: Western medicines
SR: Systematic review
MA: Meta-analysis
AMSTAR-2: Assessing the Methodological Quality of Systematic Reviews-2
GRADE: Grading of Recommendations, Assessment, Development, and Evaluation
PRISMA: Preferred Reporting Item for Systematic Reviews and Meta-Analyses
ICU: Intensive care unit
APACHE: Acute physiology and chronic health evaluation
PCT: Procalcitonin
RCT: Randomized controlled trials
WMD: Weighted mean difference
SMD: Standard mean difference
MD: Mean difference
OR: Odds ratio
RR: Relative risk.
